The article "The Impact of the COVID-19 Pandemic on the Incidence, Severity, and Management of Acute Appendicitis: A Single Center Experience in Thailand" was published in 2022. Journal: Emerg Med Int.

# The Impact of the COVID-19 Pandemic on the Incidence, Severity, and Management of Acute Appendicitis: A Single Center Experience in Thailand

**DOI:** 10.1155/2022/8324716

**Published:** 2022-11-24

**Authors:** Chompoonut Achavanuntakul, Prasit Mahawongkajit, Saritphat Orrapin, Karikarn Auksornchat, Piyapong Boonyasatid, Nichakarn Waewsri, Alisa Moriguchi, Amonpon Kanlerd

**Affiliations:** Department of Surgery, Faculty of Medicine, Thammasat University, Thammasat University Hospital, Pathumthani, Thailand

## Abstract

**Purpose:**

For more than two years since the COVID-19 pandemic, human lives have changed, including the healthcare system. Management of acute appendicitis, the most common emergency surgical disease, has been inevitably affected. This study aimed to assess the effect of the COVID-19 pandemic on the incident rate of complicated appendicitis, management, outcome, and complication of acute appendicitis. *Patients and Methods*. This study was a retrospective cohort study comparing 574 patients diagnosed with acute appendicitis before the COVID-19 outbreak and 434 patients diagnosed with acute appendicitis during the COVID-19 outbreak. Patient demographic data, type of appendicitis, type of treatment, time to surgery, length of stay, cost, and complications were collected and analyzed.

**Results:**

During the COVID-19 pandemic, the number of patients diagnosed with acute appendicitis was reduced. CT scan usage for diagnosis was increased compared to pre-COVID-19. Most patients diagnosed with acute appendicitis received operative treatment in both groups. Median time to surgery was significantly longer during the COVID-19 pandemic, 11.93 hours compared to 9.62 hours pre-COVID-19, *p*-value <0.001 (relative risk 1.5, 95% CI 1.29–1.76, *p* value 0.041). The incidence of complicated appendicitis was not higher during COVID-19. Compared to pre-COVID-19, ICU admission rate, the use of a mechanical ventilator, length of stay, and cost increased in the univariate analysis but were not statistically significant in the multivariate analyses. Other treatment complications had no statistically significant difference.

**Conclusion:**

The incidence of complicated appendicitis did not increase during the COVID-19 pandemic. The operation waiting time significantly increased but did not increase the rate of treatment complications in a well-prepared hospital system.

## 1. Introduction

Acute appendicitis is both the most common cause of abdominal pain [1] as well as surgical emergency disease worldwide [2], including in Thailand. The lifetime risk of acute appendicitis is 8.6% in males and 6.7% in females [3]. The most effective treatment is surgical appendectomy [4], while nonoperative treatment with antibiotics is an alternative method of treatment [5], especially in uncomplicated acute appendicitis. Current data show the safety of nonoperative treatment of acute appendicitis [1]; many high-quality studies and guidelines encourage nonoperative treatment with antibiotics in acute appendicitis with a good outcome, low rate of complication, and decreased length of hospital stay [6] but increased risk of recurrence (39%) in 5 years [1, 7].

The article "The Impact of the COVID-19 Pandemic on the Incidence, Severity, and Management of Acute Appendicitis: A Single Center Experience in Thailand" was published in 2022. Journal: Emerg Med Int.

Since the first case of COVID-19 was reported [8] and become a pandemic [9], the healthcare system needed to relocate resources and staff in the pandemic era. Some surgical nurses were required to leave the operating room and work in the field hospital for COVID-19. Intensive care unit (ICU) hospital beds and ventilators were preserved for COVID-19 patients. Staff had to separate into two groups: one work and one stay-at-home, alternating periodically, to minimize face-to-face contact and avoid being a COVID-19 super spreader. Elective surgery was postponed due to closed operating rooms at a maximum of 50% capacity, except for diseases that affect the quality of life such as impending rupture abdominal aorta, critical limb ischemia, or cancer [10–13]. The effect of COVID-19 impacted not only elective surgery cases but also emergency cases due to the limit of the emergency operating rooms at daytime and nighttime. Most of the cases needed to delay operations more than normal and needed to wait for the COVID-19 PCR result before going to surgery, except for extremely urgent cases such as trauma or severe peritonitis with unstable vital signs. Acute appendicitis was inevitably affected. To date, most of the literature reported the effect of COVID-19 on acute appendicitis from the beginning of the pandemic, which meant that there was a low sample size and only short-term outcomes were reported but now we have lived with COVID-19 for more than two years, so this study aims to evaluate the effect of COVID-19 on acute appendicitis in a long-term period.

## 2. Material and Methods

### 2.1. Study Population

We conducted a retrospective cohort study of adult patients with acute appendicitis who were treated at Thammasat University Hospital between January 31, 2018, and January 30, 2022. The inclusion criteria were adult patients (age at least 18-year-old) who were diagnosed with acute appendicitis by the International Classification of Diseases and Related Health problem 10th Revision (code: K35-37) and were admitted to the ward. The exclusion criteria were being unable to collect data from medical records or missing medical records, patients denied the treatment and left the hospital, patients with elective appendectomy, and patients with chronic appendicitis. Populations were divided into 2 comparable groups, pre-COVID-19 group, defined as patients in the 2 years before the in-country spreading of COVID-19 (January 31, 2018, until January 30, 2020), and during COVID-19 group, defined as patients in the 2 years after in-country spreading of COVID-19 (January 31, 2020, until January 30, 2022).

The article "The Impact of the COVID-19 Pandemic on the Incidence, Severity, and Management of Acute Appendicitis: A Single Center Experience in Thailand" was published in 2022. Journal: Emerg Med Int.

The Human Research Ethics Committee of Thammasat University (Medicine) gave approval and waived informed consent requirements, the Number Certificate of Approval is 109/2022, and the project Number is MTU-EC-SU-1-067/65. This study was registered with the Thai Clinical Trials Registry on June 15, 2022, reference number was TCTR20220615001.

### 2.2. Data Collection

The electronic medical record and chart review were conducted. Demographic data of patients including age, sex, weight, height, body mass index (BMI), underlying disease, American Association of Anesthesiologist (ASA) score, clinical presentation such as duration of self-report symptom, nausea or vomiting, right lower quadrant pain, fever, diarrhea, rebound tenderness, vital sign, laboratory data such as leukocytosis and neutrophil predominate, along with radiologic data, treatment method, operative time, time to surgery, histopathological data, type of appendicitis, length of stay, cost, and complication were obtained.

The primary objective was the incidence of complicated appendicitis during the COVID-19 outbreak compared to the pre-COVID-19 outbreak. The secondary objectives were to compare complication rate, length of hospital stay, time to surgery, and cost.

### 2.3. Statistical Analysis

All baseline characteristics and demographic data were assessed in both pre-COVID-19 and during COVID-19 period. Mean and standard deviation (SD) with Student *t*-test analysis were performed in the normal distribution group. The nonparametric test was performed by Mann–Whitney test and reported in median with interquartile range (iqr) to compare the data between pre-COVID-19 and during COVID-19 period. The *p* value <0.05 is considered statistically significant. The equality of distribution (for the data of more than 50 cases) was evaluated by histogram and the Kolmogorov–Smirnov (K–S) test. Multivariate regression analysis was performed to compare primary and secondary outcomes between pre-COVID-19 and during the COVID-19 period. All statistical analyses were performed using a STATA/SE 16.0 for Windows (Stata Corp LP, TX, USA), and *p* values <0.05 were regarded as indicating statistical significance. The study process and report followed the strengthening of the reporting of observational studies in epidemiology (STROBE) statement on reports of the cohort studies (Figure 1) [14, 15].

The article "The Impact of the COVID-19 Pandemic on the Incidence, Severity, and Management of Acute Appendicitis: A Single Center Experience in Thailand" was published in 2022. Journal: Emerg Med Int.

## 3. Results

One thousand and twenty-five patients were enrolled in this present study. Two patients refused to stay in the hospital, one in the pre-COVID-19 group and one in the during the COVID-19 group. 15 patients were excluded by exclusion criteria and missing significant data. Finally, this study consisted of 574 patients in the pre-COVID-19 group and 434 patients in the during COVID-19 group. Most general demographic data had no statistically significant difference between the two groups. However, cases diagnosed as acute appendicitis decreased in the during COVID-19 period contrary to increased airway and chronic kidney disease, which increased to ASA classification 2–4 (Table 1).

In the pre-COVID-19 period, patients presented with right lower quadrant pain, migratory pain, and fever more than during COVID-19 period. The mean body temperature was 37.29 degrees Celsius in the pre-COVID-19 group and 36.94 degree Celsius in the during COVID-19 group. Pulse rate and respiratory rate were higher in the during COVID-19 group, 92.77 beats/minute, 20.10 beats/minute in the during COVID-19 group, and 89.59 beats/minute and 19.72 beats/minute in the pre-COVID-19 group, respectively. Additionally, neutrophils predominate was higher in the during COVID-19 group (Table 1).

During the COVID-19 pandemic, patients with acute appendicitis were more likely to have a CT scan than pre-COVID-19 pandemic. The most common CT finding was fat standing followed by an enlarged appendix, more than 6 millimeters, which was more common during the COVID-19 pandemic than prepandemic. The most common treatment, surgical appendectomy, did not change but during COVID-19 period, the laparoscopic approach was higher than in pre-COVID-19. Median time to surgery was longer during COVID-19 pandemic at 11.93 hours compared to 9.62 hours in pre-COVID-19, *p* value <0.001. Operative time was similar in both groups (Table 2).

Gangrenous appendicitis was higher in the pre-COVID-19 group at 14.46% compared to 8.76% in the during COVID-19 group, *p* value 0.006. Other types of appendicitis normal, simple appendicitis, ruptured appendicitis, appendiceal abscess, and appendiceal phlegmon, were similar. The most common histopathology was appendicitis in both groups (Table 2).

Table 3 shows the outcome of the treatment. The complications pneumonia, surgical site infection, abdominal collection, ileus, anastomosis leakage, and acute kidney injury were similar in prepandemic compared to during the pandemic. However, there was a higher intensive care unit admission rate and more ventilators used during COVID-19 compared to pre-COVID-19.

The article "The Impact of the COVID-19 Pandemic on the Incidence, Severity, and Management of Acute Appendicitis: A Single Center Experience in Thailand" was published in 2022. Journal: Emerg Med Int.

No mortality case was recorded in pre-COVID-19 but one patient died of acute appendicitis during COVID-19. The death case was an 83-year-old male with underlying diseases of hypertension, heart disease, chronic kidney disease, and benign prostatic hypertrophy. The diagnosis was ruptured appendicitis. He underwent an open appendectomy, with the time to surgery being 22.78 hours. Postoperative, the patient developed surgical site infection, abdominal collection, upper gastrointestinal bleeding, coagulopathy, atelectasis then dyspnea due to pneumonia with sepsis, ileus, and non-ST-elevated myocardial infarction with volume overload and acute kidney injury. He was resuscitated, had endotracheal tube placement, and was admitted to the ICU ward, but his clinical presentation deteriorated and the patient passed away, with the total LOS being 79 days.

The mean length of hospital stay (LOS) was longer during COVID-19 compared to pre-COVID-19, along with higher expenditure during COVID-19 compared to pre-COVID-19, 23426 (17037.75, 35406.5) compared to 19395.75 (14653, 26366.5), *p* value <0.001.

Multivariate analyses of primary and secondary outcomes found no statistically significant difference in complicated appendicitis, ventilator use, ICU admission, prolonged LOS, or high cost. However, the during COVID-19 group was associated with a prolonged time to surgery of more than 10 hours with a relative risk of 1.5, 95% CI 1.29–1.76, *p* value 0.041(Table 4).

## 4. Discussion

Some previous data showed delayed presentation (>72 hours) that was significantly higher during COVID-19 than the pre-COVID-19 period, associated with higher complicated appendicitis. [7, 16, 17] We found no statistical significance of longer self-reported symptom period but there was the statistical significance of higher ASA classification, concomitant with airway and chronic kidney disease, higher pulse rate, respiratory rate, and neutrophil predominate that indicated systemic inflammatory response and more severe disease. The lower number of patients with acute appendicitis in the during COVID-19 group [18–20] may be due to the patient being afraid of in-hospital COVID-19 transmission [21, 22], so the increased threshold presenting to the hospital, a mild symptom of acute appendicitis may spontaneously regress without treatment or patients may have gone to the drug store and taken oral antibiotics by themselves and then symptoms resolved without the need of hospital treatment [18, 23–25] together with the strong government policy of stay-at-home.

The gastrointestinal presenting symptoms of COVID-19 infection mimic the symptoms of acute appendicitis [26–28] caused by multisystem inflammatory syndrome (MIS), especially in children and adolescents. Abdominal pain, nausea, vomiting, diarrhea, and loss of appetite make the diagnosis of acute appendicitis more difficult and more likely to require preoperative imaging to confirm the diagnosis. The increased rate of CT scans during the COVID-19 pandemic [20, 29] was likely due to the need to confirm the diagnosis and avoid an unnecessary operation.

The article "The Impact of the COVID-19 Pandemic on the Incidence, Severity, and Management of Acute Appendicitis: A Single Center Experience in Thailand" was published in 2022. Journal: Emerg Med Int.

The gold standard of acute appendicitis is surgical appendectomy while nonoperative treatment is an alternative method [5]. Nonoperative treatment increased during the COVID-19 pandemic [30, 31]; some national surgical guidelines [10, 32–34] and literature [23, 29, 35, 36] advocated nonoperative treatment and carefully consider a laparoscopic approach. The benefits of nonoperative treatment are no anesthetic complications and decreased staff in an operating room, therefore reducing COVID-19 exposure. In normal situations, the preferred appendectomy approach is laparoscopic more than open due to less postoperative pain, lower incidence of surgical site infection, and decreased length of hospital stay [1, 33] but, in our institutions, there is limited equipment, nurses, and surgeons skilled in laparoscopic method, as well as financial concerns because laparoscopic treatment is not covered by the universal coverage scheme. So, the mainstay of treatment is open appendectomy. At our institute, the increased rate of laparoscopic appendectomy during the pandemic was due to confounder chronological bias because the minimally invasive surgery fellowship program started in July 2021. Although laparoscopic surgery requires precautions during the COVID-19 pandemic, we had proper protective equipment and hence no staff member was infected with COVID-19 from any operation.

The time to surgery was significantly longer during the COVID-19 pandemic due to limited operating rooms and staff because the hospital policy divided staff into two groups that do not contact each other so as to limit infection if one team member became infected with COVID-19. Some operative nurses also had to leave the operating room and had a new workload to take care of COVID-19 patients. The hospital policy announced that every patient who was to undergo surgery needed to have a COVID-19 PCR test. The waiting time for the test results prolonged the time for surgery. Except for patients with emergency conditions that could not wait for test results, all staff had to do the operation in a negative pressure room and be dressed in a proper personal protective equipment suit. There was no significantly longer operative time during the pandemic. This was similar to previous literature regarding acute care surgery including acute appendicitis from Krutsri et al. [37] which found that the waiting time for surgery was significantly longer in the pandemic period compared to the previous year. Operative time and morbidity and mortality had no significant difference.

The article "The Impact of the COVID-19 Pandemic on the Incidence, Severity, and Management of Acute Appendicitis: A Single Center Experience in Thailand" was published in 2022. Journal: Emerg Med Int.

Nonoperative management with intravenous antibiotics was higher in the COVID-19 group with no increase in complication rate [29, 38, 39]. The cause of increased nonoperative treatment is likely due to the risk of perioperative morbidity-mortality in surgical patients with concomitant COVID-19 infection [40]. The PCR for the COVID-19 test result of one of the patients in the during COVID-19 group was positive, which resulted in a change of treatment plan. First, the patient was diagnosed with acute appendicitis by clinical presentation and laboratory test and it was planned to set the operating room for an open appendectomy after the report of PCR for COVID-19 test was expected to be not detected. Unfortunately, the result was detected so the surgeon decided to work up imaging by CT scan and found that the patient had an appendiceal phlegmon, so the plan of treatment changed to intravenous antibiotics alone and follow-up by clinical examination. The patient improved every day and had successful conservative treatment and was discharged from the hospital after completing isolation. Our case was similar to a case report of successful conservative management of acute appendicitis in a coronavirus disease 2019 patient from the USA [41].

Although some studies have shown higher complicated appendicitis during the COVID-19 outbreak [2, 16, 18, 21, 42, 43] along with a higher complication rate [2, 7, 35] of statistical significance, our study showed no statistically significant complicated appendicitis or complication rate during the COVID-19 outbreak. Even with significantly longer waiting times for surgery, a well-prepared healthcare system managed to maintain a standard of care during the pandemic. Similar findings from Antakia et al. [44] showed a significant increase in the radiological evaluation and an increase in nonoperative management during COVID-19 period in the United Kingdom but no significant difference in the length of hospital stays or mortality. Studies from Ganesh et al. [45] and Pringle et al. [46] also showed a significant increase in imaging investigations during the COVID-19 pandemic but no significant difference in the outcome of treatment of acute appendicitis. Zhou and Cen [42] reported on the outcome of acute appendicitis in Jiaxing, China, and reported a higher proportion of perforated appendicitis but no long-term postoperative complication was found during the pandemic. In the study from Turanli and Kiziltan [47], there was no clear increased rate of perforated appendicitis during the pandemic period (Table 5).

The article "The Impact of the COVID-19 Pandemic on the Incidence, Severity, and Management of Acute Appendicitis: A Single Center Experience in Thailand" was published in 2022. Journal: Emerg Med Int.

In univariate analysis, it was found that LOS, ICU admission, and ventilator use statistically significantly increased, possibly due to increased concomitant disease (ASA 2–4). The cost was significantly higher, which may have been caused by the expense of routine preoperative PCR COVID testing and increased LOS.

Our advice is that a preoperative CT scan is important to decrease the negative appendectomy rate and is highly recommended for patients with concomitant COVID-19 infection to avoid unnecessary operations. The waiting time for COVID-19 results is an adaptable problem for delayed time to surgery and is associated with complicated appendicitis. There should be a hospital policy and limited maximum laboratory time for testing PCR to minimize the time to surgery and provide the best outcome. We encourage patients not to hesitate and be quick to seek medical attention at a hospital if they have unusual abdominal pain because of the delayed presentation associated with higher complications.

The Covid-19 pandemic has had a negative impact on patients with acute appendicitis by increasing the time to surgery. However, complicated appendicitis, including gangrenous, rupture appendicitis, appendiceal abscess, and phlegmon, was not significantly higher during the COVID period when compared with the pre-COVID period. ICU admission, ventilator use, LOS, and cost were statistically significant in univariate analysis but not statistically significant in multivariate analyses.

At present, some countries have announced COVID-19 as an endemic, not pandemic anymore and some countries plan to do the same, so we have to adapt to a new normal everyday life and new normal medical treatment and learn to live with COVID-19. This invaluable knowledge from four years consecutive with a large population will guide the treatment of acute appendicitis in the future.

### 4.1. Limitation

This study was a retrospective study that had high selection bias and was conducted in a single large resident training university hospital that may not be generalizable to other hospitals.

### 4.2. Future Interesting Point

The characteristic of patients with acute appendicitis concomitant with COVID-19 infection will be the next interesting topic.

## 5. Conclusions

The COVID-19 pandemic has had no significant effect on complicated appendicitis but significantly delayed the time to surgery. However, it did not increase any complications of acute appendicitis under a well-prepared hospital system.

The article "The Impact of the COVID-19 Pandemic on the Incidence, Severity, and Management of Acute Appendicitis: A Single Center Experience in Thailand" was published in 2022. Journal: Emerg Med Int.

## Figures and Tables

**Figure 1:** The study flow diagram of the cohort study.

**Table 1:** Demographic data of adult patients with acute appendicitis.

	Pre-COVID-19 (*n* = 574)	During COVID-19 (*n* = 434)	*p* value
Age, mean ± SD (years)	37.46 ± 17.1	37.99 ± 17.6	0.680^*∗∗*^
Median (iqr)	33 (23, 49)	33 (23, 52)	
Gender male/female	299/275	216/218	0.465
BMI, (Kg/m^2^)	23.08 ± 4.23	23.45 ± 4.48	0.179
Underlying disease, (%)			
Hypertension	73 (12.72)	60 (13.82)	0.607
Diabetes mellitus	34 (5.92)	30 (6.91)	0.524
Heart disease	7 (1.22)	11 (2.53)	0.119
Airway disease	10 (1.74)	18 (4.15)	0.021^*∗*^
Vascular disease	10 (1.74)	10 (2.30)	0.526
Chronic kidney disease	7 (1.22)	15 (3.46)	0.016^*∗*^
Immunocompromise	12 (2.09)	9 (2.07)	0.985
ASA classification			
1	462 (80.49)	269 (61.98)	<0.001^*∗*^
2	102 (17.77)	128 (29.49)	<0.001^*∗*^
3	9 (1.57)	34 (7.83)	<0.001^*∗*^
4	0 (0)	3 (0.69)	0.046^*∗*^
5	0 (0)	0 (0)	
Sign and symptom, (%)			
Self-report symptom, (hours)			
Mean ± SD (years)	35.10 ± 49.47	36.36 ± 48.73	0.686^*∗∗*^
Median (iqr)	24 (12, 48)	24 (10, 48)	
Nausea/vomiting	355 (61.95)	283 (65.21)	0.289
RLQ pain	523 (91.27)	337 (77.65)	<0.001^*∗*^
Migratory pain	337 (58.81)	193 (44.47)	<0.001^*∗*^
Fever	268 (46.77)	130 (29.95)	<0.001^*∗*^
Diarrhea	134 (23.39)	107 (24.65)	0.640
Anorexia	250 (43.63)	198 (45.62)	0.529
Rebound tenderness	283 (49.48)	204 (47.00)	0.437
Body temperature, (°C)	37.29 ± 0.74	36.94 ± 0.68	<0.001^*∗*^
Systolic blood pressure, (mmHg)	123.06 ± 16.81	124.40 ± 17.75	0.224
Diastolic blood pressure, (mmHg)	73.18 ± 10.91	74.05 ± 12.22	0.235
Pulse rate, (beats/minute)	89.59 ± 15.76	92.77 ± 18.75	0.004^*∗*^
Respiratory rate, (beats/minute)	19.72 ± 1.45	20.10 ± 2.01	<0.001^*∗*^
Laboratory test, (%)			
Leukocytosis	405 (70.56)	311 (71.66)	0.703
Neutrophils predominate	432 (75.26)	361 (83.18)	0.002^*∗*^

ASA, American Association of Anesthesiologist; BMI, body mass index; iqr, interquartile range; RLQ, right lower quadrant; SD, standard deviation, ^*∗*^Statistically significant *p* value <0.05, ^*∗∗*^nonparametric data.

**Table 2:** Investigation, operative, and histopathology data of adult patients with acute appendicitis.

	Pre-COVID-19	During COVID-19	*p* value
Radiological investigation			
CT scan, (%)	188 (32.75)	197 (45.39)	<0.001^*∗*^
CT finding, (%)			
Fecalith	62 (32.98)	50 (25.38)	0.101
Fat standing	176 (93.2)	193 (97.97)	0.032^*∗*^
Size (more than 6 mm)	172 (91.49)	192 (97.46)	0.010^*∗*^
Perforation	46 (24.47)	45 (22.84)	0.707
Collection	49 (26.06)	33 (16.75)	0.026^*∗*^
Treatment, (%)			
Appendectomy (vs nonoperative management)	541 (94.25)	402 (92.63)	0.299
Type of appendectomy			0.028^*∗*^
Open	537 (99.26)	392 (97.51)	
Laparoscopic	4 (0.74)	10 (2.49)	
Antibiotic	214 (37.28)	182 (41.94)	0.134
Percutaneous drainage	23 (4.01)	21 (4.84))	0.522
Time to surgery, (hours)			<0.001^*∗*^,^*∗∗*^
Mean ± SD (years)	10.9 ± 6.61	13.75 ± 8.34	
Median (iqr)	9.62 (7.4, 13)	11.93 (8.5, 17)	
Operative time, (minutes)			0.269^*∗∗*^
Mean ± SD (years)	77.3 ± 44.52	78.49 ± 37.68	
Median (iqr)	68 (50, 95)	71 (55, 93)	
Type of appendicitis, (%)			
Normal	2 (0.35)	1 (0.23)	0.733
Simple appendicitis	362 (63.07)	274 (63.13)	0.982
Gangrenous appendicitis	83 (14.46)	38 (8.76)	0.006^*∗*^
Ruptured appendicitis	117 (20.38)	89 (20.51)	0.962
Appendiceal abscess	28 (4.88)	27 (6.22)	0.353
Appendiceal phlegmon	19 (3.31)	13 (3.00)	0.778
Histopathology, (%)			
Appendicitis	535 (98.89)	400 (99.50)	0.311
Malignancy	3 (0.55)	0 (0)	0.135
Normal	2 (0.37)	1 (0.25)	0.744
No appendix tissue	1 (0.18)	1 (0.25)	0.833

CT, computerized tomography; iqr, interquartile range; SD, standard deviation, ^*∗*^Statistically significant *p* value <0.05. ^*∗∗*^nonparametric data.

The article "The Impact of the COVID-19 Pandemic on the Incidence, Severity, and Management of Acute Appendicitis: A Single Center Experience in Thailand" was published in 2022. Journal: Emerg Med Int.

**Table 3:** Outcome of the treatment in adult patients with acute appendicitis.

	Pre-COVID-19	During COVID-19	*p* value
Complication, *n* (%)			
ICU admission	2 (0.35)	9 (2.07)	0.009^*∗*^
Ventilator use	1 (0.17)	8 (1.84)	0.005^*∗*^
Pneumonia	0 (0)	2 (0.46)	0.104
Surgical site infection	29 (5.05)	27 (6.22)	0.422
Abdominal collection	11 (1.92)	8 (1.84)	0.933
Ileus	13 (2.26)	12 (2.76)	0.613
Anastomosis leakage	1 (0.17)	0 (0)	0.384
Acute kidney injury	9 (1.57)	8 (1.84)	0.737
Mortality, *n* (%)	0 (0)	1 (0.23)	0.250
LOS			0.001^*∗*^,^*∗∗*^
Mean ± SD (days)	3.2 ± 2.47	4.0 ± 5.14	
Median (iqr)	3 (2, 4)	3 (2, 4)	
Expenditure, (baht)			<0.001^*∗*^,^*∗∗*^
Median (iqr)	19395.75 (14653, 26366.5)	23426 (17037.75, 35406.5)	

ICU, invasive care unit; iqr, interquartile range; LOS, length of hospital stay, ^*∗*^Statistically significant *P*-value <0.05, ^*∗∗*^nonparametric data.

**Table 4:** Multivariate analyses of primary and secondary outcomes.

	Relative risk (RR)	95% CI	*p* value
Primary outcome			
Gangrenous appendicitis	0.70	0.53–0.92	0.338
Ruptured appendicitis	1.01	0.84–1.19	0.292
Appendiceal abscess	1.14	0.86–1.51	0.979
Appendiceal phlegmon	0.94	0.61–1.44	0.772
Secondary outcome			
Prolonged time to surgery^*a*^	1.50	1.29–1.76	0.041^*∗*^
Ventilator use	2.08	1.63–2.65	0.457
ICU admission	1.91	1.43–2.55	0.420
Prolonged LOS^*b*^	1.19	1.03–1.38	0.332
High cost^*c*^	1.34	1.16–1.55	0.075

ICU, invasive care unit; LOS, length of hospital stay. ^*a*^ categorized by prolonged time to surgery by the time of patient's arrival to the operation more than 10 hours (by the median value). ^*b*^ categorized to long LOS by admission in hospital more than 3 days (by the median value). ^*c*^ categorized as the high cost of treatment by the total cost of treatment of more than 20,000 baht (by the median value). ^*∗*^ Statistically significant *p* value <0.05.

The article "The Impact of the COVID-19 Pandemic on the Incidence, Severity, and Management of Acute Appendicitis: A Single Center Experience in Thailand" was published in 2022. Journal: Emerg Med Int.

**Table 5:** Literature review of COVID-19 and acute appendicitis.

Authors (year)	Origin	Sample size	Research design	Purpose	Summary of finding
Sathik et al. [2] (2020)	India	155	Retrospective and prospective observational study	To compare the presentation, grade of presentation, and postoperative complications of AA before and during the COVID-19 pandemic	Significant increase in complicated appendicitis, LOS, and postoperative surgical site infection during COVID-19 pandemic
El Nakeeb et al. [7] (2022)	Middle east	1,945	Multicenter prospective cohort study	To compare the presentation and outcomes of patients with AA who presented during the COVID-19 pandemic and before the onset of the pandemic	Decrease in the number of patients with AA was seen along with a higher incidence of complex AA, greater use of CT scanning, and more application of NOM during the COVID-19 pandemic More postoperative complications, reoperation, and readmission during the COVID period
Javanmard-emamghissi et al. [35] (2021)	UK	500	Multicenter prospective cohort study	To determine the impact of the first weeks of the pandemic on the management of AA	Median LOS as significantly reduced in NOM group and 30 days complications were significantly higher in operative group. NOM shown to be safe and effective in the short-term, antibiotics should be considered as the first line during the pandemic and perhaps beyond
Zhou and Cen [42] (2020)	China	90	Retrospective study	To assess the efficacy of the management of AA during the COVID- 19 pandemic	Higher proportion of perforated appendicitis and chief complaint duration for perforated appendicitis was longer during COVID-19 pandemic No long-term postoperative complication was found
Zaikos et al. [43] (2021)	USA	283	Retrospective observational study	To determine the effect the early COVID-19 pandemic period had on the presentation, management, and histopathologic severity of AA	No significant change in the number of patients presenting with AA Significant increase in the incidence of perforated appendicitis decreased surgical management
Antakia et al. [44] (2021)	UK	207	Prospective cohort study	To determine the efficacy and outcomes of conservative versus surgical management of AA during the pandemic	Significant increase in radiological evaluation and conservative management during COVID-19 period For those managed operatively an open approach was preferred intraoperative findings were suggestive of delayed presentation during the COVID period without affecting the LOS and mortality
Ganesh et al. [45] (2020)	UK	96	Retrospective study	To compare the management of appendicitis and postoperative outcomes between pre- and post-COVID-19	Significant increase in imaging investigation and decrease in surgery during COVID-19 pandemic but no significant difference in the outcome
Pringle et al. [46] (2021)	UK	247	Retrospective cohort study	To compare the presentation, management, and outcomes of AA before and during the COVID-19 pandemic	No observed increase in severity of AA during the COVID-19 pandemic patients had a shorter LOS and were more likely to have imaging NOM proportionally increased with no observed change in outcomes
Turanli and Kiziltan [47] (2021)	Turkey	214	Retrospective observational study	To assess the clinical presentation and delays in diagnosing AA during the COVID-19 pandemic	No observable clear increase rate of perforated appendicitis during pandemic period

AA, acute appendicitis; LOS, length of hospital stay; NOM, non-operative management; UK, United Kingdom; USA, United States of America.

The article "The Impact of the COVID-19 Pandemic on the Incidence, Severity, and Management of Acute Appendicitis: A Single Center Experience in Thailand" was published in 2022. Journal: Emerg Med Int.

## Data Availability

The data used to support the findings of this study are included within the article.

## References

[1] Di Saverio S., Podda M., De Simone B. (2020). Diagnosis and treatment of acute appendicitis: 2020 update of the WSES Jerusalem guidelines. *World Journal of Emergency Surgery*.

[2] Sathik S. R., Karthick D., Rajmohan, Jayalal J. A. (2020). Acute appendicitis during COVID-19: changing clinical presentation and outcome. *International Journal of Health Sciences & Research*.

[3] Addiss D. G., Shaffer N., Fowler B. S., Tauxe R. V. (1990). The epidemiology of appendicitis and appendectomy in United States. *American Journal of Epidemiology*.

[4] Sartelli M., Baiocchi G. L., Di Saverio S. (2018). Prospective observational study on acute appendicitis worldwide (POSAW). *World Journal of Emergency Surgery*.

[5] Collaborative C., Flum D. R., Davidson G. H., Chen T. (2020). A randomized trial comparing antibiotics with appendectomy for appendicitis. *New England Journal of Medicine*.

[6] Yang Z., Sun F., Ai S., Wang J., Guan W., Liu S. (2019). Meta-analysis of studies comparing conservative treatment with antibiotics and appendectomy for acute appendicitis in the adult. *BMC Surgery*.

[7] El Nakeeb A., Emile S. H., AbdelMawla A. (2022). Presentation and outcomes of acute appendicitis during COVID-19 pandemic: lessons learned from the Middle East-a multicentre prospective cohort study. *International Journal of Colorectal Disease*.

[8] Guan W. J., Ni Z. Y., Hu Y. (2020). Clinical characteristics of Coronavirus disease 2019 in China. *New England Journal of Medicine*.

The article "The Impact of the COVID-19 Pandemic on the Incidence, Severity, and Management of Acute Appendicitis: A Single Center Experience in Thailand" was published in 2022. Journal: Emerg Med Int.

[9] Cucinotta D., Vanelli M. (2020). WHO declares COVID-19 a pandemic. *Acta BioMedica*.

[10] Joint guidance for surgeons (2020). *Guidance for Surgeons Working during the COVID-19 Pandemic from the Surgical Royal Colleges of the United Kingdom and Ireland*.

[11] Joint guidance for surgeons (2020). *Updated Intercollegiate General Surgery Guidance on COVID-19*.

[12] Moletta L., Pierobon E. S., Capovilla G. (2020). International guidelines and recommendations for surgery during Covid-19 pandemic: a Systematic Review. *International Journal of Surgery*.

[13] Joint Statement (2020). *Roadmap for Maintaining Essential Surgery during COVID-19 Pandemic American College of Surgeons*.

[14] von Elm E. A. D., Altman D. G., Egger M., Pocock S. J., Gøtzsche P. C., Vandenbroucke J. P. (2008). The Strengthening the Reporting of Observational Studies in Epidemiology (STROBE) statement: guidelines for reporting observational studies. *Journal of Clinical Epidemiology*.

[15] Vandenbroucke J. P. V. E. E., von Elm E., Altman D. G. (2014). Strengthening the reporting of observational studies in epidemiology (STROBE): explanation and elaboration. *International Journal of Surgery*.

[16] Orthopoulos G., Santone E., Izzo F. (2021). Increasing incidence of complicated appendicitis during COVID-19 pandemic. *The American Journal of Surgery*.

[17] Kearney D., Cahill R. A., O’Brien E., Kirwan W. O., Redmond H. P. (2008). Influence of delays on perforation risk in adults with acute appendicitis. *Diseases of the Colon & Rectum*.

[18] Chang Y. J., Chen L. J., Chang Y. J. (2022). Did the severity of appendicitis increase during the COVID-19 pandemic?. *PLoS One*.

[19] Slagman A., Behringer W., Greiner F. (2020). Medical emergencies during the COVID-19 pandemic. *Dtsch Arztebl Int*.

[20] Romero J., Valencia S., Guerrero A. (2020). Acute appendicitis during Coronavirus disease 2019 (COVID-19): changes in clinical presentation and CT findings. *Journal of the American College of Radiology*.

[21] An S., Kim H. R., Jang S., Kim K. (2022). The impact of the Coronavirus disease-19 pandemic on the clinical characteristics and treatment of adult patients with acute appendicitis. *Front Surg*.

[22] Wong L. E., Hawkins J. E., Langness S., Murrell K. L., Iris P., Sammann A. (2020). Where are all the patients? Addressing covid-19 fear to encourage sick patients to seek emergency care. *NEJM Catalyst*.

[23] Podda M., Pata F., Pellino G., Ielpo B., Di Saverio S. (2021). Acute appendicitis during the COVID-19 lockdown: never waste a crisis. *British Journal of Surgery*.

[24] Tankel J., Keinan A., Blich O. (2020). The decreasing incidence of acute appendicitis during COVID-19: a retrospective multi-centre study. *World Journal of Surgery*.

The article "The Impact of the COVID-19 Pandemic on the Incidence, Severity, and Management of Acute Appendicitis: A Single Center Experience in Thailand" was published in 2022. Journal: Emerg Med Int.

[25] Farinha H. T., Gilgien J., Di Mare L. (2021). Appendicitis and cholecystitis during the COVID-19 outbreak: a multicentre experience. *Swiss Medical Weekly*.

[26] Malbul K., Katwal S., Maharjan S., Shrestha S., Dhital R., Rajbhandari A. P. (2021). Appendicitis as a presentation of COVID-19: a case report. *Annals of Medicine and Surgery*.

[27] Abdalhadi A., Alkhatib M., Mismar A. Y., Awouda W., Albarqouni L. (2020). Can COVID 19 present like appendicitis?. *IDCases*.

[28] Martin A., Otto T., Smith T. (2021). A case of COVID-19 mimicking acute appendicitis in multi-system inflammatory syndrome. *Cureus*.

[29] English W., Habib Bedwani N., Smith C. (2021). Suspected appendicitis and COVID-19, a change in investigation and management-a multicentre cohort study. *Langenbeck’s Archives of Surgery*.

[30] Collard M., Lakkis Z., Loriau J. (2020). Antibiotics alone as an alternative to appendectomy for uncomplicated acute appendicitis in adults: changes in treatment modalities related to the COVID-19 health crisis. *Journal of Visceral Surgery*.

[31] Basamh M., Rajendiran A., Chung W. Y., Runau F., Sangal S. (2020). Management of appendicitis during the COVID pandemic: lessons from the first month of the outbreak. *British Journal of Surgery*.

[32] Brücher B. L. D. M., Nigri G., Tinelli A. (2020). COVID-19: pandemic surgery guidance. *4open*.

[33] Alemanno G., Tomaiuolo M., Peris A., Batacchi S., Nozzoli C., Prosperi P. (2020). *SAGES and EAES Recommendations Regarding Surgical Response to COVID-19 Crisis*.

[34] Association of Upper Gi Surgery of Great Britain and Ireland (2020). AUGIS Guidelines: management algorithm for patients with clinically suspected appendicitis during Covid-19 pandemic. AUGIS.

[35] Javanmard-Emamghissi H., Boyd-Carson H., Hollyman M. (2021). The management of adult appendicitis during the COVID-19 pandemic: an interim analysis of a UK cohort study. *Techniques in Coloproctology*.

[36] Ielpo B., Podda M., Pellino G. (2021). Global attitudes in the management of acute appendicitis during COVID-19 pandemic: ACIE Appy Study. *British Journal of Surgery*.

[37] Krutsri C., Singhatas P., Sumpritpradit P. (2021). Impact of the COVID-19 pandemic on the outcome, morbidity, and mortality of acute care surgery patients: a retrospective cohort study. *International Journal of Surgery Open*.

[38] Patel V. K., Ye K., In H., Scheinfeld M. H. (2021). Non-operative management for acute appendicitis during the COVID-19 pandemic does not increase the rate of complications. *Journal of Gastrointestinal Surgery*.

[39] English W., Habib Bedwani N., Smith C., Shatkar V. (2020). Investigation and management of suspected appendicitis during the COVID-19 pandemic. *British Journal of Surgery*.

The article "The Impact of the COVID-19 Pandemic on the Incidence, Severity, and Management of Acute Appendicitis: A Single Center Experience in Thailand" was published in 2022. Journal: Emerg Med Int.

[40] Collaborative C., Bhangu A., Glasbey J. C. (2020). Mortality and pulmonary complications in patients undergoing surgery with perioperative SARS-CoV-2 infection: an international cohort study. *Lancet (London, England)*.

[41] Suwanwongse K., Shabarek N. (2020). Successful conservative management of acute appendicitis in a Coronavirus disease 2019 (COVID-19) patient. *Cureus*.

[42] Zhou Y., Cen L. S. (2020). Managing acute appendicitis during the COVID-19 pandemic in Jiaxing, China. *World Journal of Clinical Cases*.

[43] Zaikos T. D., Boudiab E. M., Peshel E. C. (2021). Acute appendicitis severity during the early COVID-19 pandemic period. *Trauma Surg Acute Care Open*.

[44] Antakia R., Xanthis A., Georgiades F. (2021). Acute appendicitis management during the COVID-19 pandemic: a prospective cohort study from a large UK centre. *International Journal of Surgery*.

[45] Ganesh R., Lucocq J., Ekpete N. O. (2020). Management of appendicitis during COVID-19 pandemic; short-term outcomes. *Scottish Medical Journal*.

[46] Pringle H. C. M., Donigiewicz U., Bennett M. R. (2021). Appendicitis during the COVID-19 pandemic: lessons learnt from a district general hospital. *BMC Surgery*.

[47] Turanli S., Kiziltan G. (2021). Did the COVID-19 pandemic cause a delay in the diagnosis of acute appendicitis?. *World Journal of Surgery*.

